This article has been retracted.

# Intelligent Correction Method of Shooting Action Based on Computer Vision

**DOI:** 10.1155/2022/8753473

**Published:** 2022-07-11

**Authors:** Bo Li, Lei Wang, Hao Feng

**Affiliations:** ^1^School of Sport Sciences, Lingnan Normal Univesity, Zhanjiang 524048, China; ^2^Department of Physical Education, Tangshan Normal University, Tangshan 063000, China; ^3^Police Physical Education Department, Hebei Vocational College for Correctional Police, Shijiazhuang 050081, China

## Abstract

Aiming at the problem that the students' long-term use of nonstandard shooting action leads to poor basketball teaching effect, an intelligent correction method of shooting action based on computer vision is proposed. Combined with the principle of computer vision, the image acquisition model of basketball shooting action is constructed. The edge contour and adaptive feature segmentation of basketball images are detected, and abnormal shooting movements are recognized. The intelligent correction model of shooting action is constructed, and the intelligent correction of shooting action is realized. Finally, through experiments, it is proved that the visual analysis and intelligent correction effect of basketball shooting action are obviously better, and it can correct shooting action in real time and accurately.

## 1. Introduction

The accuracy and standard of shooting in basketball are directly related to the score, which is of great significance to the reasonable test and judgment of basketball shooting. At present, the standardized judgment of basketball shooting is lack of systematic theory. The visual analysis method is often used to modify and optimize basketball shooting [1]. The visual analysis methods of basketball shooting action are mainly divided into three categories: establish a direct topology, count the visual feature sampling points of basketball shooting action, and carry out feature classification and recognition in combination with the cloud distribution in the uniform and dense pixel space, but it is limited in practical sports.

Based on the visual analysis method of sports image based on the CT/MRus model, the action and body position of basketball shooting are a dynamic change process [2]. The model cannot automatically reconstruct the standardization process of basketball shooting, and the correction effect of target shape is not good. Combining the above two methods, the template registration method is used for visual analysis, the step-by-step three-dimensional structure model in the process of basketball shooting is constructed, and the action orientation and amplitude are optimized by the iterative method to improve the reliability of the action [3]. The key to this method lies in the construction of basketball shooting action template shape and the selection of standardized action correction constraint rules. In the visual analysis of basketball shooting action, we need to give consideration to accuracy and real time.

In order to improve the standard judgment level of basketball action, a standardized judgment method of basketball action based on computer vision is proposed. Through the edge contour detection and feature segmentation of shooting image, the nonstandard shooting action is recognized, and the intelligence correction of shooting action is realized. Its performance is analyzed through a specific application example.

## 2. Intelligent Correction Method of Shooting Action

### 2.1. Basketball Shooting Image Acquisition Model

Based on the basketball shooting video information of computer vision, the target detection algorithm is used to obtain the human body detection frame area of basketball players for computer vision. Then, based on the human-computer vision algorithm, the detected players are computer vision, and the joint point information of basketball players is extracted. Finally, based on the calculation method of joint point offset angle change in three-dimensional space, this article compares the joint point information of basketball players with that of standard action, obtains the difference between learners' action and standard action, and makes a quantitative and qualitative analysis on whether learners' action is standard or not [4, 5]. At the same time, it gives the corresponding suggestions for the improvement of action posture to help learners correct actions and improve the effect of basketball learning. The flow chart is shown in Figure 1.

The motion similarity calculation method based on human joint point extraction mainly includes the following steps: firstly, the position information of human joint points in the standard image and the target image is extracted. Then standardize the actions on the two pictures, convert their coordinates, and overlay them into the same coordinate system [6]. The offset calculation calculates the direction and length difference of each joint point after standardization and infers and calculates the angle difference between the joint point of the target image and the standard action in three-dimensional space. According to the calculation of the deviation angle between the learner's action and each joint point of the standard action, the quantitative index of action similarity is designed to calculate the similarity between the basketball action and each joint point of the standard action [7]. Select the joint with the lowest score, correct the coordinate of the corresponding joint position information in the standard action image again, and restore the standard action corresponding to the joint position with nonstandard action to the target image through coordinate change, so as to obtain the corresponding action correction suggestions [8]. Assuming that the computer vision model marks the spatial rotation of basketball shooting action, at multiple points in the space of basketball shooting, it is obtained that the shape coordinate of shooting action under the initial deformation is:

(1) $$\begin{array}{c} X={\left(x_{i0},x_{i1},\ldots ,x_{i\left(n-1\right)},y_{i0},y_{i1},\ldots ,y_{i\left(n-1\right)}\right)}^{T}. \end{array}$$

The width of the whole characteristic image of the basketball court is *x*_*i*(*n* − 1)_ and the height is *y*_*i*(*n* − 1)_. The three-dimensional spatial characteristic image of basketball shooting is divided into several subblocks by using the grid model. The sampling image of basketball shooting action has 2 on the grid surface *x*_*ij*_′, *y*_*ij*_′. Two-pixel points, extract the density characteristics of sampling points and get the mean squared error between the standardized feature points (*x*_*ij*_, *y*_*ij*_) of shooting action:

(2) $$\begin{array}{c} {\text{err}}_{ij}=\frac{1}{N}-X\sum_{i=1}^{N}\sqrt{{\left(x_{ij}^{\prime }-x_{ij}\right)}^{2}+{\left(y_{ij}^{\prime }-y_{ij}\right)}^{2}}, \end{array}$$

where *n* is the total number of evenly distributed grids of the image. Considering all the pixel feature points of *n* spatial positions, the difference error vector of basketball players in shooting, lifting, and holding is:

(3) $$\begin{array}{c} p_{j}^{i}=\frac{1}{X}\sum_{j=0}^{n-1}{\text{err}}_{ij}-\frac{1}{n}. \end{array}$$

According to the degree of motion, the 17 joint points obtained are divided into 2 categories: the first category is the left and right shoulder joints and left and right hip joints with a small range of motion, which are defined as static joint points [9]. The second category is the rest of the joint points, whose motion range is relatively large, which is defined as active joint points. The static joint points defined in this article are mainly used to locate and determine the zoom ratio, so as to better compare the position of human joints between the target image and the standard image [10]. According to the two types of joint points defined, first take the left shoulder joint point in the target image as the reference position, and then superimpose it on the target image with relevant node information on the premise that all joint points in the standard image remain unchanged, so that the left shoulder joint points of the standard image and the target image coincide, so as to realize the first coordinate correction [11]. After the second coordinate correction, the joint point *P* is expressed as:

(4) $$\begin{array}{c} d=p_{j}^{i}+p_{6}^{i+1}-p_{6}^{i}, \end{array}$$

where *i* is the picture number; *j* is the number of joint points; 6 is the number of left shoulder joint points. Then, the Euclidean distance of the defined static joint points (left and right shoulder joint points and left and right hip joint points) is taken as the shoulder width and hip width of the human body, respectively [12]. Taking the ratio of the sum of shoulder width and crotch width of the target image and the standard image as the standardization basis, the connecting line between the joint points in the target image is scaled in equal proportion, and the coordinates of the corresponding joint points are corrected to obtain the second coordinate correction key point *P* of the standardization process, expressed as:

(5) $$\begin{array}{c} k=\frac{d\left(p_{6}^{i},p_{7}^{i}\right)+d\left(p_{12}^{i},p_{13}^{i}\right)}{d\left(p_{6}^{i+1},p_{7}^{i+1}\right)+d\left(p_{12}^{i+1},p_{13}^{i+1}\right)},\\ p_{j}^{i\prime }=p_{j}^{i}+k\left[p_{j}^{i}-f\left(p_{j}^{i}\right)\right]. \end{array}$$

The number is the number of joint points of the right shoulder, left arm, and right arm, respectively; *f*(*p*) represents the joint point connected with the joint point; *d*(*p*_1_, *p*_2_) represents the Euclidean distance between point *p* and point *p*_2_. After the second correction of joint point standardization, the offset of the above 8 joint points is compared and calculated. When the limb has a back and forth offset in space, the two-dimensional projection length of the limb on the picture will change, so the back and forth offset angle *p*_*k*_ of the limb in space can be deduced by using the length information of the limb:

(6) $$\begin{array}{c} p_{id}=\frac{180}{\pi }\arccos\frac{d\left(p_{k}^{i+1},f\left(p_{k}^{i+1}\right)\right)}{d\left(p_{k}^{i},f\left(p_{k}^{i}\right)\right)}, \end{array}$$

where *K* is the joint number and *P* is the center point corresponding to the joint. Thus, the pixel sampling and feature analysis of the three main position spaces of basketball players are realized. The computer graphics processing method is used to make the standardized judgment of basketball shooting action in the interactive scene. The modeling process is shown in Figure 2.

With the formation of clear action image and the establishment of correct action concept, through visual and auditory information feedback, students gradually establish the proprioception of muscle activities in imitation and trial, and the excitation and inhibition of nerve center are gradually improved and accurate in time and space, initially forming the action skill of in situ one-handed shoulder shooting, but at this time, the action is not coordinated and coherent enough, and it is easy to be disturbed by new differences or strong stimuli [13–18]. Therefore, in the differentiation stage, we should also pay attention to avoid the generation and correction of nonstandard actions. In the process of correcting errors and removing redundant actions, in addition to visual and auditory information feedback, special attention should be paid to the application of positional, tactile, and proprioceptive information feedback, for example, for the wrong actions such as elbow abduction, insufficient elbow lifting and arm extension, stiff fingers, excessive wrist flexion, backward shoulder, and dry twisting after the ball is released [19]. The feedback and enhancement of proprioceptive information can be strengthened by means of assistance (i.e., hand handle) to help lift the elbow and arm, resistance (i.e., holding the elbow joint with a hand) to remind him not to abduct too much, and repeated unarmed imitation exercises, so as to improve the coordination of his whole body force [20]. Through the feedback of multichannel sensory information, promote the further improvement of differentiation inhibition, correct wrong movements, and successfully master the complete one-handed shoulder shooting skills [4, 21–25].

### 2.2. Recognition of Shooting Error Characteristics

In the process of basketball, the image analysis is carried out in combination with the human body dynamics model [26]. When the basketball is shooting, there *v*_*id*_(*t*) is a positive motion intensity distribution. With the rotation of the basketball in the air and entering the basket frame, the probability density function of the position distribution of the ball in the air after it is released during basketball shooting is as follows:

(7) $$\begin{array}{c} P\left(I\right)=\omega v_{id}\left(t\right)+\text{cr}\left(p_{id}-x_{id}\left(t\right)\right), \end{array}$$

where cr represents the error correction weighting in the motion coordinate system. Adaptive error correction is carried out in the frame of pixel *ω*, and the standardized error correction switching motion equation of basketball shooting action is obtained through viewpoint switching

(8) $$\begin{array}{c} \frac{\partial u\left(x,y;t\right)}{\partial t}=\frac{f\left(p\right)}{P\left(I\right)-d}-v_{id}\left(t\right). \end{array}$$

This article analyzes the structure of motor skills from the perspective of computer vision and puts forward the control system model of motor skills [27–29]. This model regards motion as a complete computer vision system composed of a receptor system, the central processing function, and an effector system [30, 31]. The model emphasizes the role of the central processing function. It checks and corrects the input information through the sensory-motor program, and then controls the activity of the effector system to cause a certain motor response. Feedback plays an important role in this process (see Figure 3).

According to the process in Figure 3, the characteristics of shooting error are identified, which provides a basis for the next step of shooting action correction.

### 2.3. Intelligent Correction of Shooting Action

In basketball shooting, the posture and speed of the wrist in the inner angle are *J*, respectively. The action torque of the player's upper limb is decomposed into two forces through the characteristics, which are *θ*, *θ* ∈ *R*. Under the computational vision, image feature acquisition is used for visual segmentation, and the edge contour detection differential equation of visual image is obtained as follows:

(9) $$\begin{array}{c} {\dot{p}}_{e}=J\left(\theta \right)-\frac{\partial u\left(x,y;t\right)}{\partial t}{\dot{\xi }}^{T}\dot{\theta }, \end{array}$$

where $\dot{\xi }$ is the Jacobian matrix of the arm for basketball shooting. According to the acquisition model of the visual image of basketball shooting action, the kinematics solutions of direction, landing point, and rotation after basketball shooting are obtained as follows:

(10) $$\begin{array}{c} \gamma ={\dot{p}}_{e}+\left(I-J\right){\dot{\xi }}^{T}P\left(I\right). \end{array}$$

Let the contour line of the shooting image in the visual coordinate system be *σ*, the configuration of the motion feature image is unknown, the scale of edge contour detection and adaptive feature segmentation is *u*, and *kl* is the visual region threshold of the basketball shooting action body [32]. Because there are many body parts of athletes during shooting, the image edge amplitude information is decomposed into multiple grid feature samples. *C* represents the corner information of evenly distributed grid vertices *ϖ* and the corner points of shooting error are calibrated [33, 34]. After sampling the error points of shooting action, it is fed back to the computer for visual analysis and action correction. The estimated value of corrected shooting displacement is as follows:

(11) $$\begin{array}{c} p\left(x,y;t\right)=C\varpi -\sigma \nabla u+kl. \end{array}$$

Take the reference characteristic image of correct shooting action as a Gaussian vector with scale 1, and calculate the diameter of grid model:

(12) $$\begin{array}{c} D=p\left(x,y;t\right)\left(\max_{i\in N_{w}}\left(\gamma \right)-\min_{i\in N_{w}}\left(\gamma \right)\right). \end{array}$$

According to the above process, it is the most direct link to obtain the action posture of sports participants [35, 36] and build a virtual environment landscape. Through the three-dimensional reconstruction of the light and shade, shadow, focal length, and other passive clues in the preprocessed image, the limitation of the system on the scale and position of the modeled scene can be reduced to the greatest extent, as shown in Figure 4.

Aiming at the application of shooting action correction, after getting the three-dimensional reconstruction model provided by the system, the sports participants can intuitively see the virtual results of their own actions. So far, the correction of shooting action is realized.

## 3. Analysis of Experimental Results

The hardware environment of the experimental platform is the CPU is Intel Core I3 processor 3.30 GHz, the memory is 4 GB DDR3, and the sampling resolution of the visual image of basketball shooting action is 320 × 240. A group of basketball shooting action visual image simulation data expresses a basketball shooting action. There are 100 test sample image sets in each shooting action mode, and there are 1024 in the basketball shooting action visual image database × 1000 test sets, establish a simplified visual analysis model of basketball shooting action with solid works, import the analysis data into ADAMS software for image processing and visual analysis, and make a standardized judgment on basketball shooting action. After 40 students are randomly divided into groups, experiment with the two groups of students for two months. Then, the shooting action of the control group is not specially corrected in class at ordinary times, while the experimental group pays special attention to the correction of its shooting action, and stipulates that the in situ one-handed shoulder shooting is the correct shooting action. The data of the experimental sample is shown in Figure 5:

The measurement of shooting hit rate adopts fixed-point shooting in the free-throw area, each person throws 3 groups, each group throws 10 times, and the average of the 3 groups is taken as the shooting hit rate. The shooting percentage data of 20 players in the control group and the experimental group before training, 2 weeks of training, 4 weeks of training, 6 weeks of training, and 8 weeks of training were statistically processed, and the average was obtained for comparison. Data statistics are shown in Table 1:

Significance of normative evaluation and detection of one-handed shoulder shot during basketball marching: normative data acquisition method showing technical actions during the whole shooting process: one teacher counts and whistles with a stopwatch, and the other teacher records and observes together. Finally, take the average score of the two teachers as 5 as the student's performance measurement method: the tester shoots on the free-throw line now, starts timing at the same time, and grabs the backboard after shooting on the free-throw line, starts from the right side, dribble with the left hand to the center line, then turn around and lay up with the right hand. After the ball hits the basket, grab the backboard, dribble with the right hand to the left-center line, turn around and shoot with the left hand. Experimental requirements: if the free-throw line fails to shoot, you can continue to run the basket. When the running basket fails to shoot, you need to make up the basket until you hit (see Tables 2 and 3 for details).

According to a series of tests conducted on all students in the control group before the experiment, the students may have no detailed action concept and proficiency in the standardization of the overall technical action. So, after a round of study, jump shot *P* (0.05 has a significant difference, and the average number has increased by 2 compared with that before the experiment: there is no significant difference between the standardization of jump shot and the speed of running basket *P* > 0.05: there is a significant difference between the standardization of running basket *P*=0.05, and the average score has also increased compared with that before the experiment. Based on the analysis of the above results, we can conclude that the standardization of jump shot and running basket has been significantly improved after learning the traditional teaching mode: while the speed of jump shot and running basket has been improved in the traditional teaching mode. There is no significant difference after learning, which leads to the result that the traditional teaching mode has no special training for the standardization of jump shot and running basket. Some experimental results of basketball posture comparison and correction suggestions according to the algorithm proposed in this article are shown in Tables 4 and 5.

The computer vision analysis process of 20 shooting movements is averaged, and the adaptive correction and action standardization judgment are carried out in the three-dimensional space of shooting movements. The results are shown in Table 6:

It can be seen from Table 6 that the algorithm in this article can correct the shooting deviation in real-time and accurately, realize adaptive real-time correction, and guide basketball shooting training. Two groups of teaching classes were randomly selected from my teaching parallel classes for teaching verification and comparison. One group is the teaching class of general physical education and the other group is the teaching class of basketball special course. The two groups set up one verification class and one comparison class, respectively, with 21 people in each class. In order to ensure the reliability and validity of the research, the students in the selected class were predicted for shooting error correction before verification, and there was no significant difference in the prediction results (*P* > 0.05), The teaching of in situ one-handed shoulder shooting technology is conducted for a total of 3 weeks and 6 class hours. The information feedback is applied to the teaching of the verification class, the conventional teaching is conducted in the comparison class, and the error correction test comparison of the same standard is conducted after the practical teaching. The comparison results are shown in Tables 7 and 8.

From the comparison results of classroom teaching verification research in the table, it can be seen that the error correction scores of the verification class are better than those of the comparison class, and there is a significant difference (*P* < 0.05). It can be seen that the application of information feedback in basketball technology teaching is helpful to form the correct dynamic shaping of shooting technology and improves the teaching quality and efficiency of basketball technology.

## 4. Discussion

Through communication with coaches, this article compares the action completion of excellent athletes, and analyzes the irrationality of their own behavior, so as to correct it in future training. In addition, using the established perfect function expansion system, we can establish an automatic comparison interface to automatically compare the movement changes in a cycle and the movement comparison between ourselves and other excellent athletes, and assist in the manual analysis of movement elements. Firstly, the technical action images of elite athletes in related fields are collected for three-dimensional reconstruction, and the complete three-dimensional posture data of these athletes are obtained. Secondly, according to the three-dimensional pose data extraction technology provided in this article, the effective feature information of three-dimensional pose data of elite athletes is quantified; Thirdly, take mining information as the system standard, and finally establish the standard model database to enrich the standard action model in the system database. Under this technical condition, the more technical actions entered by excellent athletes, the more they can help later users learn more excellent actions, so as to optimize their sports actions. After comparing with the actions in the database, the system will score the user's action score according to the scoring system in the competition, which is convenient for the user to obtain the evaluation results more directly. In the teaching of shooting, the height of the basketball is reduced, so that students can effectively adjust the radian when shooting. Students can compare the results of different shooting radians. At the same time, students can also practice various control abilities of the ball when shooting, and understand the relationship between various factors when shooting, such as the relationship between shooting speed, shooting angle, and the angle of entering the basket, so that students can form a correct understanding of the essence of shooting. In order to guide their practice, it is precisely because the students themselves participate in the learning of shooting. Through their own perception and adjustment of the movement, the students' cognition of the shooting technical movement is more accurate, which is conducive to the learning of shooting technology. The time to correct mistakes is very important. If it is late, it is hard to correct, if it is early, there are many mistakes, and we cannot start. Therefore, we should seize the opportunity of correction according to the different stages of students' mastery of motor skills. In the early stage of physical education learning, the main purpose of students is to experience the feeling of sports. At this time, due to the students' insufficient understanding of sports technology and lack of profound understanding, there will be many wrong behaviors and redundant behaviors. Therefore, the requirements for students' sports technology at this stage should not be too high. In classroom teaching, students' common wrong behaviors can be corrected, and students' personal problems can be guided by personal guidance. In the second stage of mastering motor skills, that is, the stage of improvement and improvement, students' nervous system and muscle system begin to coordinate, and errors begin to reduce. At this time, teachers' requirements for students are gradually improved, especially the key links and key links of sports technology, which require students to do well and accurately. In the consolidation stage of sports skills, we should focus on the details of sports technology and improve the quality of sports technology.

## 5. Conclusions

The accuracy and standard of basketball shooting are directly related to the score. The reasonable judgment of basketball shooting action is an important factor to improve the level of basketball training. Therefore, a standardized judgment method of basketball shooting action based on computer vision is proposed. The simulation experiment shows that there is a significant difference when the jump shot *P* is less than 0.05, and the average number is 2 more than that before the experiment: there is no significant difference between the jump shot standardization and the running basket speed *P* > 0.05; there is a significant difference between the running basket *P*=0.05 standardization. The following conclusions can be drawn: the computer vision analysis of basketball shooting action using this method can correct the shooting deviation in real time and accurately. The standardized judgment time of fixed-point shooting is shorter and the accuracy is higher than that of sports shooting. Whether it is fixed-point shooting or sports shooting, the adaptive real-time correction efficiency of shooting action is good, which can effectively guide basketball shooting training.

## Figures and Tables

**Figure 1:** Motion feature extraction process of human joint points.

**Figure 2:** Standardized judgment process of basketball shooting action under computer vision.

**Figure 3:** Error identification process of the dominant effector motion system.

**Figure 4:** Error correction and correction of basketball image.

**Figure 5:** The experimental sample data.

**Table 1:** Statistics of subjects.

Number of people	Frequency	Before training		Training for 2 weeks		Training for 4 weeks		Training for 6 weeks		8 weeks of training	
		Control group (%)	Experience group (%)	Control group (%)	Experience group (%)	Control group (%)	Experience group (%)	Control group (%)	Experience group (%)	Control group (%)	Experience group (%)
20	10 × 3	17.7	16.5	18.8	15.1	20.3	27.6	23.5	34.5	25.5	40

**Table 2:** Normative evaluation of one-handed shoulder shot during basketball progress.

Achievement	Score	Evaluation criterion
Excellent	8–10 points	The action is correct and skilled, shooting a shot, and dribbling with left and right hands
Good	6–7 points	The action is correct and skilled, and the shooting is a hit
Pass	3–5 points	The action is basically correct and skilled
Fail	1–2 points	Incorrect and unskilled movements

**Table 3:** Technical difference test of the control group before and after the experiment.

	Before experiment	After the experiment	*T*	*P*
Number of jump shots	5.85 ± 2.31	8.09 ± 1.76	−0.295	0.002
Standardization of jump shot	5.89 ± 1.51	5.50 ± 1.70	−1.02	0.162
Basket running speed	72.81 ± 8.56	72.81 ± 10.09	0.15	1.00
Basket running standardization	4.37 ± 1.76	5.51 ± 1.71	−0.25	0.015

**Table 4:** Judgment of whether the learner's shooting action is standard by this method.

Visual angle	Number of samples	Correct number	Accuracy (%)
Positive	193	176	91.19
Side	33	26	78.79
Back	55	48	87.27

**Table 5:** Calculation results of shooting action similarity and posture correction suggestions based on computer vision.

Group	Overall similarity	Attitude suggestion
Group 1	0.7607	Improved left elbow posture
Group 2	0.9209	Improved right elbow posture
Group 3	0.7521	Improved left elbow posture
Group 4	0.8652	Improved left knee posture
Group 5	0.8898	Improved left elbow posture
Group 6	0.7851	Improved right leg posture
Group 7	0.7785	Improved right elbow posture
Group 8	0.8752	Improved right elbow posture

**Table 6:** Analysis results of basketball shooting action transformation judgment.

Mode	Number of vertices	Number of feature reconstruction triangles	Total sampling points	Judgment time (ms)	Smoothing time (ms)	Judgmentaccuracy (%)
Fixed point	4322	11093	922	12.11	212	98.11
Motion	2433	28293	1212	23.08	322	97.73

**Table 7:** Comparison results of error correction of one-handed shoulder shot with traditional methods (*n* = 21).

Class	*n*	*x*	*s*	*t*	*p*
Validation team	21	82.763	4.752	—	—
Comparison class	2	77.668	6.07	12.98	<0.05

**Table 8:** Comparison results of error correction of one-handed shoulder shot in this method (*n* = 21).

Class	*n*	*x*	*s*	*t*	*p*
Validation team	21	86.192	6.072	—	—
Comparison class	2	81.145	7.518	3.352	<0.05

## Data Availability

The data used to support the findings of this study are available from the corresponding author upon request.
